# Machine Learning with Quantum Seagull Optimization Model for COVID-19 Chest X-Ray Image Classification

**DOI:** 10.1155/2022/6074538

**Published:** 2022-03-30

**Authors:** Mahmoud Ragab, Samah Alshehri, Nabil A. Alhakamy, Wafaa Alsaggaf, Hani A. Alhadrami, Jaber Alyami

**Affiliations:** ^1^Information Technology Department, Faculty of Computing and Information Technology, King Abdulaziz University, Jeddah 21589, Saudi Arabia; ^2^Centre of Artificial Intelligence for Precision Medicines, King Abdulaziz University, Jeddah 21589, Saudi Arabia; ^3^Mathematics Department, Faculty of Science, Al-Azhar University, Naser City 11884, Cairo, Egypt; ^4^Pharmacy Practice Department, Faculty of Pharmacy, King Abdulaziz University, Jeddah, Saudi Arabia; ^5^Pharmaceutics Department, Faculty of Pharmacy, King Abdulaziz University, Jeddah, Saudi Arabia; ^6^Center of Excellence for Drug Research and Pharmaceutical Industries, King Abdulaziz University, Jeddah 21589, Saudi Arabia; ^7^Mohamed Saeed Tamer Chair for Pharmaceutical Industries, King Abdulaziz University, Jeddah 21589, Saudi Arabia; ^8^Medical Laboratory Technology Department, Faculty of Applied Medical Sciences, King Abdulaziz University, P.O. BOX 80402, Jeddah 21589, Saudi Arabia; ^9^Molecular Diagnostic Lab, King Abdulaziz University Hospital, King Abdulaziz University, P.O. BOX 80402, Jeddah 21589, Saudi Arabia; ^10^Special Infectious Agent Unit, King Fahd Medical Research Center, King Abdulaziz University, P.O. BOX 80402, Jeddah 21589, Saudi Arabia; ^11^Diagnostic Radiology Department, Faculty of Applied Medical Sciences, King Abdulaziz University, Jeddah 21589, Saudi Arabia; ^12^Imaging Unit, King Fahd Medical Research Center, King Abdulaziz University, Jeddah 21589, Saudi Arabia

## Abstract

Early and accurate detection of COVID-19 is an essential process to curb the spread of this deadly disease and its mortality rate. Chest radiology scan is a significant tool for early management and diagnosis of COVID-19 since the virus targets the respiratory system. Chest X-ray (CXR) images are highly useful in the effective detection of COVID-19, thanks to its availability, cost-effective means, and rapid outcomes. In addition, Artificial Intelligence (AI) techniques such as deep learning (DL) models play a significant role in designing automated diagnostic processes using CXR images. With this motivation, the current study presents a new Quantum Seagull Optimization Algorithm with DL-based COVID-19 diagnosis model, named QSGOA-DL technique. The proposed QSGOA-DL technique intends to detect and classify COVID-19 with the help of CXR images. In this regard, the QSGOA-DL technique involves the design of EfficientNet-B4 as a feature extractor, whereas hyperparameter optimization is carried out with the help of QSGOA technique. Moreover, the classification process is performed by a multilayer extreme learning machine (MELM) model. The novelty of the study lies in the designing of QSGOA for hyperparameter optimization of the EfficientNet-B4 model. An extensive series of simulations was carried out on the benchmark test CXR dataset, and the results were assessed under different aspects. The simulation results demonstrate the promising performance of the proposed QSGOA-DL technique compared to recent approaches.

## 1. Introduction

Coronavirus disease (COVID-19) should be diagnosed in early stages in order to reduce the spread of virus and prevent further complications. With the increasing spread of COVID-19 cases, on a day-to-day basis across the globe, the limitation of the present diagnosis tool imposes challenges in managing and curbing the outbreak. Global researchers have conducted vigorous research to develop efficient diagnosis procedures and speed up the development of treatments and vaccine [1]. In general, three diagnostic procedures are widely employed such as medical imaging, blood tests, and viral tests [2]. One of the most widely employed viral tests that is identified as the gold-standard for detecting COVID-19 is Reverse Transcription Polymerase Chain Reaction (RT-PCR) which is employed as first-line screening tool. However, a number of researchers found that the experiment results achieved a sensitivity between 50 and 62% only [3]. This reveals the fact that first RT-PCR results could be attained as negative also. Therefore, in order to validate the accuracy of the experimental diagnoses, many RT-PCR experiments are conducted on a 14-day period of observation. In other words, an RT-PCR negative result for a suspicious COVID-19 case is taken into account as True Negative, if there is no positive RT-PCR result after running screening tests during the 14-day period of observation. Practically, this frustrates the patient diagnosed with COVID-19 and stresses the already-exhausted healthcare infrastructure of most of the nations due to lack of sufficient RT-PCR kits and qualified personnel [4].

As per the literature, chest X-rays (CXR) were employed as a first-line diagnosis tool in Italy and several countries [5]. Radiology scans can be run to detect the condition of the lungs and the patient's distinct phase of recovery/illness in an efficient manner [6]. Radiologists have observed a range of abnormalities present in radiology scan reports of COVID-19 patients. In recent years, deep learning, observed as the fundamental component of enhancing Artificial Intelligence technology, was stated to have considerable diagnosis accuracy, in medical imaging, for automated diagnosis of lung disease. It exceeded human level performances on ImageNet classification tasks with one million images to train in 2015 and further displayed dermatologist level performances on the classification of skin lesions in 2017. It further produced outstanding results in terms of screening lung cancer in 2019 [7].

In general, a radiologist's manual screening process may bring bias or wrong diagnoses and increases the possible risk of lost diagnoses for minuscule lesions. Therefore, health professionals such as radiotherapists gain excellent benefit out of emerging Artificial Intelligence (AI) methods in computer-aided COVID-19 diagnostics. Artificial Intelligence (AI) and advanced software, in the field of healthcare image analyses, have directly assisted the healthcare professionals in fighting this novel coronavirus. These systems offer effective and high-quality diagnosis result and drastically reduces manpower requirement [8]. Recently, machine learning and deep learning, the two main fields of AI, have forayed into healthcare applications commonly. Deep learning-based support system is established in the diagnosis of COVID-19 using X-ray and CT scan samples. Few schemes have been proposed according to the pretrained models using transfer learning, whereas some methods have been presented with a personalized network [9]. Data science and machine learning, though being different domains, have been brought together and are dynamically employed in different stages such as prognosis, diagnosis, outbreak forecasting, and prediction for COVID-19. However, almost all of the DL-based techniques, used in disease diagnosis, require annotating the lesion, particularly for the disease diagnoses in CT volume. Annotating the lesion of COVID-19 incurs heavy cost, time, and effort for the radiotherapist which prevents efficient curbing of the disease. COVID-19 has rapidly spread to global nations, and there is a huge shortage for radiotherapists. Therefore, conducting COVID-19 diagnosis using DL models is of great significance for the community.

The current study focuses on the design of a new Quantum Seagull Optimization Algorithm with DL-based COVID-19 diagnosis model, named QSGOA-DL technique. Besides, the proposed QSGOA-DL technique involves the design of EfficientNet-B4 as a feature extractor, whereas the hyperparameter optimization process is carried out by the QSGOA technique. Moreover, the classification process is performed by a multilayer extreme learning machine (MELM) model. In order to showcase the supremacy of the proposed QSGOA-DL technique, a wide range of experimental analyses was conducted on benchmark test CXR dataset and the results were assessed under several aspects.

The rest of the paper is organized as follows: Section 2 reviews the literature; Section 3 discusses the proposed model; Section 4 validates the performance of the proposed model; at last, Section 5 concludes the study.

## 2. Related Works

Roy et al. [10] presented a new deep network acquired from the spatial transformer network. This network can predict the disease's seriousness rate concurrently based on input frames and offer positioning of pathological artefact in a weakly supervised manner. Additionally, the authors presented a novel methodology according to the uninorm for aggregation of efficient frame scores at a video level. At last, advanced deep methods were validated to estimate the pixel-level segmentation of COVID-19 imaging biomarker. In [11], a matrix profile technique was presented to detect the abnormalities in CT scan image through two stages. Abnormality Severity Score (CT-SS) was evaluated, and the variance of CT-SS between the COVID-19 CT image and non-COVID-19 CT image was examined. A sparse abnormality mask was evaluated and used for penalizing the pixel value of all the images. The abnormality-weighted images were utilized later for training the benchmark DenseNet DL model to differentiate COVID-19 CT from non-COVID-19 CT image. In this study, the authors applied the VGG19 model as a baseline model for comparison purposes.

Sakib et al. [12] proposed a feasible and effective DL-CRC framework for distinguishing COVID-19 from other abnormalities (for example, pneumonia) and usual case with high precision. Exclusive datasets were developed from four open sources with PA chest sight of X-ray information for pneumonia, COVID-19, and usual case. The presented DL-CRC frameworks leveraged the DARI model for COVID-19 data by adaptively using GAN and GAD models. Kaur et al. [13] proposed expert models on the basis of deep feature and PF-BAT enhanced PF-FKNN classifiers to diagnose the novel coronavirus. In the presented method, the feature is extracted from the FC layer of transfer-learned MobileNetv2 and FKNN training. The hyperparameter of FKNN is fine-tuned with the help of PF-BAT algorithm.

Singh and Singh [14] proposed an automatic approach to diagnose COVID-19 from chest X-ray images. The study proposed an enhanced depth-wise CNN model to analyze the chest X-ray image. Wavelet decompositions were used in this study to integrate multiresolution analyses in the network. The frequency subbands, attained from the input image, were fed into the network to identify the disease. The networks were developed to predict the class of input image as either COVID-19 or normal or viral pneumonia.

Li et al. [15] proposed a new method for efficient and effective training of COVID-19 classification network with less number of COVID-19 CT exams and a record of negative samples. Specifically, new self-supervised learning methods were introduced to extract the features from negative sample and COVID-19-positive samples. Next, two types of soft labels (“diversity” and “difficulty”) were made for a negative sample by calculating the earth mover distance between COVID-19 features and negative samples, where the data “value” of the negative sample could be measured. Shamsi et al. [16] presented a deep uncertainty-aware TL architecture for COVID-19 recognition using healthcare image. Four common CNNs, including InceptionResNetV2, VGG16, ResNet50, and DenseNet121, were initially used in this study to extract the deep features from CT and X-ray images. Later, feature extraction was accomplished using distinct ML and statistical modelling methods to identify COVID-19 cases.

Wu et al. [17] developed a new JCS system to execute explainable and real-time COVID-19 chest CT diagnoses. In order to train these JCS systems, the authors created a large-scale COVID-19 Segmentation and Classification (COVID-CS) dataset containing 144,167 chest CT images collected from 400 COVID-19 persons and 350 negative samples. A total of 3,855 chest CT images, collected from 200 persons, were annotated to fine-grained pixel-level label of opacification, i.e., improved attenuation of lung parenchyma. Han et al. [18] proposed an AD3D-MIL model in which a person-level label is allocated to a 3D chest CT scan image that is viewed as a bag of instance. AD3D-MIL could semantically create deep 3D instances by following the probably diseased region. Furthermore, AD3D-MIL employs an attention-based pooling method for 3D instances so as to provide insight to every instance that contributes toward bag labels. Finally, AD3D-MIL learns Bernoulli's distribution of bag-level label for easily available learning.

## 3. The Proposed Model

In this study, a novel QSGOA-DL technique is presented to detect and classify COVID-19 using CXR images. The presented QSGOA-DL technique encompasses different operational stages such as preprocessing, EfficientNet-B4-based feature extraction, QSGO-based hyperparameter optimization, and MELM-based classification.  Figure 1 illustrates all the processes involved in the proposed QSGOA-DL model. The design of QSGO technique assists in optimal selection of hyperparameter values of EfficientNet-B4 model.

### 3.1. Preprocessing

In the presented model, the images undergo preprocessing through two ways such as data augmentation and image resizing. The augmentation technique generates the perturbed versions of the available images. Scaling, rotations, and other affine conversions are commonly used herewith. It is generally carried out to increase the size of the dataset and provide effective training to the deep learning model on different types of images. Besides, the 2D array (*x*-axis and *y*-axis) of the image of X-data (size of 512 × 512) is normalized for pixel values between 0 and 255 and stored from PNG format with the help of OpenCV library. All the preprocessed images measure 512 × 512 and have three channels.

### 3.2. EfficientNet-B4-Based Feature Extraction

In this stage, the preprocessed CXR images are passed onto EfficientNet-B4 technique and generate a useful set of feature vectors. Here, the CNN is directed towards an acyclic graph. This network is able to learn extremely nonlinear functions too. Neurons are the fundamental unit inside a CNN. All the layers, in a CNN, are made up of many neurons. These neurons are hooked together, i.e., the output of neuron from layer *l* becomes the input of neuron at layers *l*+1, as given in the following equation:

(1) $$\begin{array}{c} a^{\left(l+1\right)}=f\left(W^{\left(l\right)}a^{\left(l\right)}+b^{\left(l\right)}\right), \end{array}$$

where *W*^(*l*)^ represents the weight matrix of layers *l*, *b*^(*l*)^ denotes bias term, and *f* indicates the activation function. The activation for layer *l* is represented as *a*^(*l*)^. In order to train a CNN, it is important to learn *W* and *b* for all the layers, so the cost functions are minimalized [19]. Generally, assume a training set {(*x*^(1)^,  *y*^(1)^),   …, ( *x*^(*m*)^,  *y*^(*m*)^)} with *m* training example; weight *W* and bias *b* should be defined since they minimize the cost, i.e., the differences between the preferred output  *y* and actual output *f*_*W*,*b*_(*x*). The cost functions for individual training examples are determined as follows:

(2) $$\begin{array}{c} J\left(W,\;b;x,\;y\right)=\frac{1}{2}{\left\|h_{W,b}\left(x\right)-y\right\|}^{2}, \end{array}$$

where *h*(*x*) represents the activation of final layer. Minimization process is iteratively performed by following the gradient descent method. This method involves the computation of partial derivatives of cost functions with regard to weight and updates the weight consequently. A single iteration of gradient descent updates the variables *W* and *b* as follows:

(3) $$\begin{array}{c} W^{\left(l\right)}=W^{\left(l\right)}-\alpha \frac{\partial }{\partial W^{\left(l\right)}}J\left(W,\;b\right),\\ b^{\left(l\right)}=b^{\left(l\right)}-\alpha \frac{\partial }{\partial b^{\left(l\right)}}J\left(W,\;b\right). \end{array}$$

The BP model is employed in the computation of a partial derivative of cost function. Each FC has a hidden unit interconnected to each input unit. This increases the numbers of connections to extreme levels, while at the same time, it can also handle high-dimension information such as images. When the image size is assumed to be its dimensions, then the process of interconnecting every input pixel to all the neurons incurs heavy computation cost. An image as small as 100 × 100 pixel requires 10^4^ × *N* connection at the input layer, in which *N* represents the number of neurons at the initial layer. The convolution layer allows the construction of a sparse connection by assigning parameters through neurons. In comparison with the FC layer, the convolution layer has fewer parameters. So, it can be trained easily. It is derived at the cost of small reduction in the performance. The widely employed CNN for image detection includes convolutional and FS layers too. This network is frequently called as a deep network.

In DL training procedure models, expansion of network width, intensification of network depth, and improvement of input image solutions are the most widely employed methods to improve the precision of the models. Even though previous works such as ResNet and WideResNet proved the supremacy of the abovementioned approaches, it is important to balance each dimension in network resolution or width or depth so that the balance could be attained by scaling all the dimensions at a constant ratio. Tan presented the EfficientNet models that could produce appropriate effects on the extension of resolution, depth, and width of the networks and later attain a better performance. Initially, the researchers could portray CNN as a function: *Y*_*i*_=*F*_*i*_(*X*_*i*_), in which *F*_*i*_ represents the operator (*op*), *Y*_*i*_ indicates the tensor of output, and *X*_*i*_ signifies the input tensor of shape 〈*H*_*i*_, *W*_*I*_, *C*_*i*_〉, where  *C*_*i*_, *H*_*i*_ , and *W*_*i*_ denote the numbers of channels of an input image, height, and width. A CNN could be determined as a sequence of layers: Net=*F*_*k*_⊙…⊙*F*_2_⊙*F*_1_(*X*_1_)=⊙_*j*=1…*k*_F_j_(*X*_1_). In actual application procedure, the CNN layers are generally employed at many phases, where every phase uses a similar network framework. Hence, it is determined as follows [20]:

(4) $$\begin{array}{c} \text{Net}=\underset{i=1\ldots s}{⊙}F_{i}^{L_{i}}\left(X_{\langle H_{i},W_{i},C_{i}\rangle }\right), \end{array}$$

where *F*_*i*_^*L*_*i*_^ represents the layer *F*_*i*_ which is continued *L*_*i*_ time in a phase *i* and 〈*H*_*i*_, *W*_*I*_, *C*_*i*_〉 represents the height, width, and numbers of channels of input tensor *X* of a layer *i*.  Next, the standard CNN design mostly focuses on identifying an optimum layer framework *F*_*i*_. However, according to the predetermined *F*_*i*_ baseline network framework, model scaling mostly extends the resolution (*H*_*i*_,  *W*_*i*_), length (*L*_*i*_), and width (*C*_*i*_) of the networks. In the meantime, model scaling overcomes the implementation problems for a novel resource constraint by setting *F*_*i*_. They could also examine *L*_*i*_, *C*_*i*_, *H*_*i*_,  and *W*_*i*_ distinctly for all the layers because it is a sample design space. EfficientNet stresses that each layer should be uniformly scaled by a constant ratio to reduce the design space. The target is to considerably enhance the precision of the models in the provided resource constraint environment since it is considered as an optimization problem:

(5) $$\begin{array}{c} \underset{d,w,r}{\max}\text{Accuracy }\left(\text{Net}\left(d,\;w,\;r\right)\right),\\ \text{s. t. Net }\left(d,\;w,\;r\right)={⊙}_{j=1\ldots k}{\hat{F}}_{i}^{d\cdot {\hat{L}}_{i}}\left(X_{\langle r\cdot {\hat{H}}_{i},r\cdot {\hat{W}}_{i},w\cdot {\hat{C}}_{i}\rangle }\right),\\ {\text{Memory }\left(\text{Net}\right)\leq \text{terget}}_{-}\text{memory,}\\ \text{FLOPS }\left(\text{Net}\right)\leq \text{ terget\_flops}, \end{array}$$

where *w*, *d*, and *r* represent the coefficients employed to scale the width, depth, and resolution of the network; $\hat{F_{i}},{\hat{L}}_{i},\hat{H_{i}},\hat{W_{i},}\text{ and }{\hat{C}}_{i}$ represent the predetermined parameters in the baseline network. Next, a novel compound scaling technique, using a compound coefficient  *ϕ*, is employed for uniform expansion of depth and width of the network as follows:

(6) $$\begin{array}{c} \text{depth}:\;d=\alpha^{\phi },\\ \text{width}:w=\beta^{\phi },\\ \text{resolution}:r=\gamma^{\phi },\\ \text{s. t}.\;\alpha \cdot \beta^{2}\cdot \gamma^{2}\approx 2,\\ \alpha \geq 1,\;\beta \geq 1,\;\gamma \geq 1\;, \end{array}$$

where *α*, *β*, and *γ* are constants. Amongst others, *ϕ* represents a stated value that determines how much resource is valid for expanding the models, whereas *α*, *β*, and *γ* determine the allocation method of extra resources to resolution, width, and depth of the network correspondingly. Also, there is a certain relationship between the FLOPS of a standard convolutional op and *d*, *w*^2^, and *r*^2^. When the depth of network doubles, then FLOPS doubles as well. However, when the network resolution/width doubles, FLOPS quadruples. Since convolutional ops frequently control the computational costs in the CNN, the CNN is expanded with equation (7) which accurately increases the overall FLOPS as (*α* · *β*^2^ · *γ*^2^)^*ϕ*^.  At last, scaling models does not alter the layer operator *F*_*i*_ in the predetermined baseline networks. Therefore, it is crucial to have a baseline network in place. EfficientNet, a novel mobile-size baseline network, is proposed with multiobjective neural framework which enhances both FLOPS and accuracy. The fundamental component consists of squeeze and excitation optimization and mobile-inverted bottleneck MBConv.

### 3.3. Hyperparameter Optimization

The QSGOA technique is deployed for optimal selection of hyperparameters involved in the EfficientNet-B4 model. In line with this, the performance gets boosted. Seagulls (scientific term: *Larus minutus*) are one amongst the coastal birds that started inhabiting the planet before 30 million years. They exist nearly everywhere in the world. With large wings, seagulls' hind legs have evolved so that they can travel in water too. Though fish is cited as the major food source for seagulls, they also consume amphibians, reptiles, moles, earthworms, and insects. In other terms, seagulls are omnivorous. They are considered as intelligent birds, while the average life span of seagulls is between 10 and 15 years. Generally, they live as a swarm and have a unique behaviour at the time of migration.

Migration is the movement of birds to the south during fall and to north during moving/spring from the ground to the height or from coast-coast to endure the winter condition and get wealthy food source with adequate amount of ease. This migration phenomenon of seagulls, which is a seasonal behaviour, is taken into account since they migrate everywhere to achieve a wide range of food sources to gain sufficient energy [21]. The procedure is given as follows:

- Migration starts when swarms of seagulls started travelling towards north/south. In order to evade collision, their primary position is made distinct from one another.
- One of the benefits from this swarm's experience is that they attempt to travel in the direction of optimal survival so as to achieve the minimum cost value.

In general, seagulls attack the migrating birds on the sea. This phenomenon occurs as a spiral-shaped behaviour at the time of attack. Seagull models for SGO are deliberated through the following points. The migration behaviour simulates the mobility of seagull swarms towards the position. For this purpose, three conditions must be fulfilled.

Collision avoidance: in order to evade the collisions amongst the neighboring seagulls, the models are determined as further parameter *A* to update the novel position of the deliberated seagull (search agents):

(7) $$\begin{array}{c} \overset{⟶}{P}=A\times {\overset{⟶}{p}}_{c}\left(i\right),\\ i=0,1,2,\;\ldots \;,\text{ Max}\left(i\right), \end{array}$$

where ${\overset{⟶}{P}}_{N}$ describes the location that avoids colliding with other search agents, ${\overset{⟶}{p}}_{c}\left(i\right)$ represents the location of the candidates in their current iteration (*i*), and *A* describes the movement behaviour of searching agents in their searching region which is also modelled as follows:

(8) $$\begin{array}{c} A=f_{c}-\left(i\times \left(\frac{f_{c}}{\text{Max}\left(i\right)}\right)\right),\; \end{array}$$

where *i* describes the iteration and *f*_*c*_ represents the frequency control of parameter *A* in the range of [0,  *f*_*c*_].

(i) With another neighbors' experience: after avoiding the collision from the neighbor, the candidate progresses in the direction of optimal neighbors (optimal solutions).
  (9) $$\begin{array}{c} {\overset{⟶}{d}}_{e}=B\times \left(\overset{⟶}{P}\left(i\right)-{\overset{⟶}{p}}_{c}\left(i\right)\right), \end{array}$$
where ${\overset{⟶}{d}}_{e}$ describes the position ${\overset{⟶}{p}}_{c}\left(i\right)$ of candidate towards an optimal fitness candidate ${\overset{⟶}{p}}_{b}\left(i\right)$. The coefficient *B* is an arbitrary value which makes the trade-off between exploration and exploitation phases. *B* is attained as follows:
  (10) $$\begin{array}{c} B=2\times A^{2}\times R. \end{array}$$
Let *R* describe the arbitrary values between zero and one.
(ii) Migration towards optimal solutions (search agents): at last, search agents upgrade their location according to the optimal solutions as follows:
  (11) $$\begin{array}{c} {\overset{⟶}{D}}_{e}=\left|{\overset{⟶}{P}}_{N}+{\overset{⟶}{d}}_{e}\right|,\; \end{array}$$
where ${\overset{⟶}{D}}_{e}$ describes the variance between optimal costs and seagulls.

At the time of migration, seagulls change the attack speed and angle frequently. The location of seagulls can be retained in the air by using their wings and weight. During attack procedure, the seagull moves in a spiral direction in air in *x*, *y*, and *z* plane by

(12) $$\begin{array}{c} X=r\times cos\left(t\right),\\ y=r\times \text{sin}\left(t\right),\\ Z=r\times t, \end{array}$$

where *t* describes arbitrary values in the range between 0 and 2*π* and*r* denotes the radius of spiral turn as per the following formula:

(13) $$\begin{array}{c} r=\alpha \times e^{\beta t}, \end{array}$$

where *e* describes the natural logarithm base and *α* and *β* represent the shapes of the spiral. The novel positions of the seagull are upgraded as follows:

(14) $$\begin{array}{c} {\overset{⟶}{P}}_{c}\left(i\right)=\left({\overset{⟶}{D}}_{e}\times \hat{x}\times \hat{y}\times \hat{z}\right)+{\overset{⟶}{P}}_{b}\left(i\right), \end{array}$$

where ${\overset{⟶}{P}}_{c}\left(i\right)$ keeps the optimal result. In order to improve the exploration abilities of SGO algorithm, QSGOA is designed including quantum computing.

Bit is the smallest unit of data from digital computers which demonstrates either 0 or 1 at a particular time, while *Q*-bit or quantum bit has achieved minimum unit of data from quantum computing. All *Q*-bits are capable to exist in the range of 0, 1, or a group of combined states simultaneously. This is named as superposition. *Q*-bit is referred to as a pair of numbers (*α*, *β*), in which the values of |*α*|^2^ and |*β*|^2^ signify the probabilities of determining the *Q*-bit from the states 0 and 1 correspondingly. The state of *Q*-bit is projected as follows:

(15) $$\begin{array}{c} |\psi =\alpha |0+\beta |1. \end{array}$$

All the *Q*-bits must fulfill the normalization formula given as follows:

(16) $$\begin{array}{c} {\left|a\right|}^{2}+{\left|\beta \right|}^{2}=1. \end{array}$$

In quantum computer, a separate *q* is signified as the order of *nQ*-bits as follows [22]:

(17) $$\begin{array}{c} q=\left[q_{1},q_{2},\ldots ,q_{n}\right]=\left[\begin{array}{ccc} \begin{array}{c} \alpha_{1}\\ \beta_{1} \end{array}| & \begin{array}{cc} \begin{array}{c} \alpha_{1}\\ \beta_{2} \end{array}| & \cdots \end{array} & |\begin{array}{c} \alpha_{n}\\ \beta_{n} \end{array} \end{array}\right]\;. \end{array}$$

When a quantum state's performance is detected, it collapses toward the single state. The observation procedure of *Q*-bit *i* is carried out as follows:

If rand. (0,1) < (*α*_*i*_)^2^

Then. *f*_*i*_=0

Else. *f*_*i*_=1

In quantum computer, the order of quantum functions is implemented to update the values to *Q*-bits from all the individuals. This results in adherence of the upgraded *Q*-bits as in equation (20). *Q*-gate is the most quantum function to update *Q*-bits. There exist different *Q*-gates such as NOT gate, controlled NOT gate, rotation gate, Hadamard gate, *x*-gate, *y*-gate, and *z*-gate. In major analysis, the rotation *Q*-gate is utilized over other Q-gates. The rotation *Q*-gate *U*(Δ*θ*_*i*_) can be determined as follows:

(18) $$\begin{array}{c} U\left(\Delta \theta_{i}\right)=\left[\begin{array}{cc} \cos\left(\Delta \theta_{i}\right) & -\sin\left(\Delta \theta_{i}\right)\\ \sin\left(\Delta \theta_{i}\right) & \cos\left(\Delta \theta_{i}\right) \end{array}\right], \end{array}$$

where Δ*θ*_*i*_ refers to the rotation angle of *Q*-bit *i* near 0/1 state. The state of *Q*-bit *i* at time *t* gets upgraded as follows:

(19) $$\begin{array}{c} \left[\begin{array}{c} \alpha_{i}\left(t+10\right)\\ \beta_{i}\left(t+1\right) \end{array}\right]=U\left(\Delta \theta_{i}\right)\left[\begin{array}{c} \alpha_{i}\left(t\right)\\ \beta_{i}\left(t\right) \end{array}\right]\;. \end{array}$$

### 3.4. Image Classification

In this final stage, the derived set of features is fed into MELM classifier to allot appropriate class labels to the test CXR images. In the basic forms of SLFN, Huang et al. presented ELM to enhance the training speed of the work and later extended the hypotheses of ELM from neurons hidden node to another hidden node. Sample training can be expressed by {*x*_*i*_,  *t*_*i*_}_*i*=1_^*n*^, where *n* represents the training sample, *x*_*i*_ indicates the input of *ith* sample using *m* dimension. Furthermore, *t*_*i*_ denotes the output of *ith* instance. Later, the input vector  *x* is assumed to be the output of SLFN using *L* hidden node, and it is expressed as follows:

(20) $$\begin{array}{c} f\left(x\right)=\overset{L}{\underset{i=1}{\sum }}\beta_{i}h_{i}\left(x\right)\\ =h^{T}\left(x\right)\beta , \end{array}$$

where *h*(*x*)=[*h*_1_(*x*) ⋯ *h*_*L*_(*x*)]^*T*^ represents the hidden output and *β*=[*β*_1_ ⋯ *β*_*L*_]^*T*^ indicates the output weight. Given the output of *n* training, the sample could be estimated by zero error and is given as follows:

(21) $$\begin{array}{c} H\beta =t, \end{array}$$

where *H*=[*h*(*x*_1_) ⋯ *h*(*x*_*n*_)]^*T*^ signifies the hidden output matrix [23]. The output weight *β* solutions involve a linear formula, while such solutions might be equal to mitigation of training errors, namely, min*Hβ* − *t*. The optimum approximation of output weight might be denoted as Moore–Penrose generalized inverse *H*^†^:

(22) $$\begin{array}{c} \hat{\beta }=H^{†}t. \end{array}$$

In general, orthogonal projection is employed to resolve the generalized inverse *H*^†^. If *H*^*T*^*H* is nonsingular, *H*^†^=(*H*^*T*^*H*)^−1^*H*^*T*^, or if *HH*^*T*^ is nonsingular, *H*^†^=*H*^*T*^(*HH*^*T*^)^−1^.

MELM is a multilayer NN in which multi-ELM-AEs are stacked together, where *X*^(*i*)^=[*x*_1_^(*i*)^,   ⋯ , *x*_*n*_^(*i*)^]; let *x*_*k*_^(*i*)^ be the *i*th data depiction for input *x*_*k*_, *k*=1 to *n*. Assume Λ^(*i*)^=[*λ*_1_^(*i*)^,   ⋯ ,  *λ*_*n*_^(*i*)^] denotes the *i*th transformation matrix, in which *λ*_*k*_^(*i*)^ denotes the transformation vectors employed in depiction learning regarding *x*_*k*_^(*i*)^. Based on this, *B* replaces with Λ^(*i*)^, where *T* is replaced by *X*^(*i*)^ correspondingly [24]:

(23) $$\begin{array}{c} H^{\left(i\right)}\Lambda^{\left(i\right)}=X^{\left(i\right)}. \end{array}$$

Let *H*^(*i*)^ be the output matrix of *i*th hidden layer with regard to *X*^(*i*)^, and Λ^(*i*)^ is resolved as follows:

(24) $$\begin{array}{c} \Lambda^{\left(i\right)}={\left(H^{\left(i\right)}\right)}^{T}{\left(\frac{I}{C}+H^{\left(i\right)}{\left(H^{\left(i\right)}\right)}^{T}\right)}^{-1}X^{\left(i\right)}. \end{array}$$

Next,

(25) $$\begin{array}{c} X^{*}=g\left(X^{\left(i\right)}{\left(\Lambda^{\left(i\right)}\right)}^{T}\right), \end{array}$$

where *χ*^*∗*^ represents the final depiction of *X*^(1)^.*X*^*∗*^ is employed as the hidden layer outputs to estimate the output weights *β*^*∗*^ and *β*^*∗*^ which are evaluated by

(26) $$\begin{array}{c} \beta^{*}={\left(X^{*}\right)}^{†},\\ T={\left(X^{*}\right)}^{T}{\left(\frac{I}{C}+X^{*}{\left(X^{*}\right)}^{T}\right)}^{-1}T. \end{array}$$

## 4. Results and Discussion

The proposed model was simulated using Python 3.6.5 tool on a benchmark CXR image dataset [25]. The results were investigated under varying sizes of training and testing datasets.  Figure 2 illustrates a few sample images considered for the study.

Figure 3 portrays the confusion matrices generated by the QSGOA-DL technique on test data with different training/testing data. Figure 3(a) depicts the confusion matrix produced by the proposed QSGOA-DL technique on training/testing of 80 : 20. The figure exhibits that the QSGOA-DL technique classified 3218 images as COVID-19 and 3219 images as healthy samples. Meanwhile, Figure 3(b) showcases the confusion matrix developed by QSGOA-DL manner on training/testing of 70 : 30. The figure shows that the QSGOA-DL algorithm outperformed compared to others and classified 3214 images as COVID-19 and 3215 images as healthy ones. Eventually, Figure 3(c) illustrates the confusion matrix generated by the QSGOA-DL algorithm on training/testing of 60 : 40. The figure demonstrates that the proposed QSGOA-DL methodology classified 3209 images as COVID-19 and 3212 images as healthy.

Table 1 shows the overall classification results attained by the QSGOA-DL technique under different training/testing data sizes. The results demonstrate that the proposed QSGOA-DL technique accomplished the maximum classification outcomes on all training/testing sizes. For instance, with a training/testing data size of 80 : 20, the QSGOA-DL technique resulted in a precision of 0.9984, sensitivity of 0.9981, specificity of 0.9984, accuracy of 0.9983, F-score of 0.9983, and MCC of 0.9966. Moreover, with a training/testing data size of 70 : 30, QSGOA-DL manner resulted in a precision of 0.9972, sensitivity of 0.9969, specificity of 0.9972, accuracy of 0.9971, F-score of 0.9971, and MCC of 0.9941. Furthermore, with a training/testing data size being 60 : 40, the proposed QSGOA-DL method produced a precision of 0.9963, sensitivity of 0.9953, specificity of 0.9963, accuracy of 0.9958, F-score of 0.9958, and MCC of 0.9916.

Figure 4 illustrates the accuracy graph plotted based on the results from the QSGOA-DL technique on the applied training/testing data size of 80 : 20. The figure reports that both training and testing accuracies got increased with an increase in epoch count. It got saturated after a maximum epoch count. It is also observed that the training accuracy got considerably higher than the testing accuracy.

Figure 5 exemplifies the loss graph plotted on the basis of results from the QSGOA-DL technique on the applied training/testing data size of 80 : 20. The figure states that both training and testing losses got heavily reduced with an increase in epoch count and got saturated after a maximum epoch count. It is noticed that the training loss is lower than the testing accuracy.

Figure 6 showcases the accuracy graph plotted based on QSGOA-DL method results on the applied training/testing of 70 : 30. The figure describes that both training and testing accuracy values got increased with an increase in epoch count and got saturated after a maximal epoch count. It is also detected that the training accuracy got significantly enhanced to the testing accuracy.

Figure 7 demonstrates the loss graph plotted based on the analysis results of QSGOA-DL method on the applied training/testing of 70 : 30. The figure indicates that both training and testing losses got increased with a higher epoch count and got saturated after a superior epoch count. It is also observed that the training loss was lesser than the testing accuracy.

Figure 8 demonstrates the results from accuracy graph analysis of QSGOA-DL algorithm on the applied training/testing of 60 : 40. The figure states that both training and testing accuracy values get enhanced with an increase in epoch count and attained saturation after a high epoch count. From the results, it can be inferred that the training accuracy is noticeably superior to the testing accuracy.  Figure 9 represents the loss graph analysis plot for the presented QSGOA-DL technique on applied training/testing of 60 : 40. The figure showcases that both training and testing losses turn into minimum value with a superior epoch count and gets saturated after an increased epoch count. It can be observed that the training loss got established and was lesser than the testing accuracy.

Finally, a detailed comparative study was conducted between the proposed QSGOA-DL technique and other recent approaches, and the results are shown in Table 2 and Figures 10 and 11 [26]. By examining the results in terms of precision, it is evident that DHL-2, ResNet-1, and ResNet-2 techniques attained a minimal precision of 97%, 97%, and 97%, respectively. Likewise, DHBL, DHL-1, and TL-ResNet-2 techniques accomplished moderate precision values of 98%, 98%, and 98%, respectively. Though TL-RENet-1 produced a near-optimal precision of 99%, the proposed QSGOA-DL technique gained a high precision of 99.80%.

Besides, with respect to sensitivity, it is clear that the models such as TL-RENet-1, ResNet-1, and ResNet-2 have obtained the least possible sensitivity of 97%, 97%, and 97%, respectively. Likewise, DHL-1, TL-ResNet-2, and DHL-2 techniques have accomplished moderate sensitivity values of 98%, 98%, and 99%, respectively. However, DBHL produced a near-optimal sensitivity of 99%, whereas the presented QSGOA-DL methodology attained a superior sensitivity of 99.80%. At the same time, by examining the results in terms of specificity, DHL-2, ResNet-1, and ResNet-2 techniques attained the least specificity values, namely, 97%, 97%, and 97%, respectively. In line with this, DHBL, DHL-1, and TL-ResNet-2 systems accomplished moderate specificity values of 98%, 98%, and 98%, respectively. TL-RENet-1 achieved a near-optimal specificity of 99%, while the projected QSGOA-DL algorithm reached the maximum specificity of 99.80%.

On the other hand, by inspecting the results in terms of accuracy, ResNet-1, ResNet-2, and TL-RENet-1 methods attained the least accuracy values of 97.21%, 97.21%, and 98.06%, respectively. Likewise, TL-ResNet-2, DHL-1, and DHL-2 methodologies too accomplished moderate accuracy values of 98.14%, 98.14%, and 98.29%, respectively. Though DBHL resulted in a near-optimal accuracy of 98.53%, the proposed QSGOA-DL manner accomplished a superior accuracy of 99.83%. The abovementioned results imply that the proposed QSGOA-DL technique outperformed the existing methods with a maximum precision of 99.80%, sensitivity of 99.80%, specificity of 99.80%, accuracy of 99.83%, F-score of 99.80%, and MCC of 99.70%. Therefore, the proposed model can be utilized as a proper tool to diagnose COVID-19 using CXR images.

## 5. Conclusion

In this study, a novel QSGOA-DL technique is presented to detect and classify COVID-19 using CXR images. The proposed QSGOA-DL technique encompasses different operational stages such as preprocessing, EfficientNet-B4-based feature extraction, QSGO-based hyperparameter optimization, and MELM-based classification. The design of QSGO technique assists in the optimal selection of hyperparameter values of EfficientNet-B4 model. In order to showcase the supremacy of the proposed QSGOA-DL technique, a wide range of experimental analyses was conducted on benchmark test CXR dataset. The results were assessed under several aspects. The simulation results demonstrate the promising performance of QSGOA-DL technique than the existing approaches. In future, the performance of QSGOA-DL technique can be validated using computed tomography (CT) scan images in the diagnosis of COVID-19.

## Figures and Tables

**Figure 1:** Overall process of the QSGOA-DL model.

**Figure 2:** Sample images.

**Figure 3:** Confusion matrix analysis results of the QSGOA-DL model.

**Figure 4:** Accuracy graph analysis of the QSGOA-DL model on training/testing (80 : 20).

**Figure 5:** Loss graph analysis of the QSGOA-DL model on training/testing (80 : 20).

**Figure 6:** Accuracy analysis results of the QSGOA-DL model on training/testing (70 : 30).

**Figure 7:** Loss analysis results of the QSGOA-DL model on training/testing (70 : 30).

**Figure 8:** Accuracy graph analysis of the QSGOA-DL model on training/testing (60 : 40).

**Figure 9:** Loss graph analysis of the QSGOA-DL model on training/testing (60 : 40).

**Figure 10:** Comparative analysis results of the QSGOA-DL model under different measures.

**Figure 11:** Accuracy analysis results of the QSGOA-DL model against existing approaches.

**Table 1:** Results of the analysis of QSGOA-DL model against different training/testing datasets.

Measures	Precision	Sensitivity	Specificity	Accuracy	F-score	MCC
Training/testing (80 : 20)	0.9984	0.9981	0.9984	0.9983	0.9983	0.9966
Training/testing (70 : 30)	0.9972	0.9969	0.9972	0.9971	0.9971	0.9941
Training/testing (60 : 40)	0.9963	0.9953	0.9963	0.9958	0.9958	0.9916
**Average**	**0.9973**	**0.9968**	**0.9973**	**0.9971**	**0.9971**	**0.9941**

**Table 2:** Comparative analysis results of the QSGOA-DL model with different measures.

Methods	Precision	Sensitivity	Specificity	Accuracy	F-score	MCC
DBHL	98.00	99.00	98.00	98.53	98.00	97.00
DHL-2	97.00	99.00	97.00	98.29	98.00	97.00
DHL-1	98.00	98.00	98.00	98.14	98.00	96.00
ResNet-2	97.00	97.00	97.00	97.21	97.00	94.00
TL-ResNet-2	98.00	98.00	98.00	98.14	98.00	96.00
ResNet-1	97.00	97.00	97.00	97.21	97.00	94.00
TL-RENet-1	99.00	97.00	99.00	98.06	98.00	96.00
QSGOA-DL	99.80	99.80	99.80	99.83	99.80	99.70

## Data Availability

Data sharing is not applicable to this article as no datasets were generated during the current study.
